# Effect of Health Belief Model Education on Increasing Cognition and Self-Care Behaviour among Elderly Women with Malignant Gynaecological Tumours in Fujian, China

**DOI:** 10.1155/2021/1904752

**Published:** 2021-10-07

**Authors:** Chenyin Liu, Xianjing Chen, Mengli Huang, Qun Xie, Qiaoming Lin, Siai Chen, Danfeng Shi

**Affiliations:** Department of Gynecology, Fujian Maternity and Child Health Hospital, Affiliated Hospital of Fujian Medical University, Fuzhou 350001, Fujian, China

## Abstract

**Objective:**

This study evaluated the effect of a health belief model (HBM) educational intervention on the self-perception of and complications related to disease in elderly gynaecological malignancy patients.

**Methods:**

This randomized controlled trial was conducted at the Fujian Maternal and Child Health Hospital, China. A total of 301 women aged 60 years and older who were diagnosed with gynaecological malignancies from January 2019 to August 2020 were recruited. Participants were randomly divided into the HBM education and basic nursing groups. The participants in the HBM education group received perioperative rehabilitation education based on the HBM, and the participants in the basic nursing group received routine basic nursing. Rehabilitation training compliance, psychological resilience, psychological flexibility, self-efficacy, self-care ability, and lower extremity deep venous thrombosis (LEDVT) incidence were assessed before and after the intervention.

**Results:**

Thirty-three women were excluded based on the exclusion criteria, and 268 participants were eventually included and randomly divided into two groups: 134 participants in the HBM education group and 134 participants in the basic nursing group. Before HBM education, there were no significant differences in the mean scores of psychological resilience (50.43 ± 3.29 vs. 50.55 ± 2.29, *P* = 0.738), psychological flexibility (48.98 ± 3.45 vs. 49.29 ± 3.59, *P* = 0.465), self-efficacy (26.49 ± 5.26 vs. 26.29 ± 6.41, *P* = 0.781), or rehabilitation training compliance (28.4% vs. 27.8%, *P* = 0.922) between the two groups. After HBM education, the scores of training compliance (80.6% vs. 30.1%, *P* < 0.001), psychological resilience (55.47 ± 5.01 vs. 50.46 ± 2.62, *P* < 0.001), psychological flexibility (56.53 ± 4.51 vs. 49.13 ± 3.62, *P* < 0.001), self-efficacy (30.79 ± 4.56 vs. 26.41 ± 6.37, *P* < 0.001), self-care knowledge (43.36 ± 7.60 vs. 34.05 ± 6.99, *P* < 0.001), self-concept (29.57 ± 5.67 vs. 20.11 ± 3.86, *P* < 0.001), self-care responsibility (27.54 ± 5.09 vs. 20.86 ± 4.53, *P* < 0.001), and self-care skills (34.51 ± 5.62 vs. 21.62 ± 5.64, *P* < 0.001) were higher in the HBM education group than those in the basic nursing group. Additionally, the incidence of LEDVT was lower in the HBM group than that in the basic nursing group (2.2% vs. 8.3%, *P* = 0.027).

**Conclusion:**

This study indicated that perioperative HBM education can improve the cognition and self-care ability of elderly gynaecological malignancy patients and reduce postoperative complications.

## 1. Introduction

In recent years, the incidence of cervical cancer, endometrial cancer, and ovarian cancer in China has increased substantially [1]; in particular, with the gradual extension of the average life span of humans, the number of elderly patients with gynaecological malignancies has increased rapidly [1]. Elderly female patients, especially elderly patients with gynaecological malignancies, have a relatively high incidence of perioperative complications due to their poor physical function, wide scope of operation, and adverse psychological effects [2]. It was reported that the incidence of postoperative complications in elderly patients with malignant gynaecological tumours can reach more than 30%, and the incidence of lower extremity deep venous thrombosis (LEDVT) accounts for more than one-third of these complications [3]. Therefore, it is essential to implement interventions to reduce the poor prognosis of elderly patients with gynaecological malignancies.

Data show that many elderly patients with gynaecological malignancies die not from the disease itself but from unawareness of their own health and unhealthy lifestyle factors [4]. The memory, psychological resilience, cognitive ability, and athletic ability of elderly patients are generally declining, causing their self-care ability and rehabilitation compliance to decrease [4–6]. Therefore, it is particularly important to pay attention to the cognitive function and health education of elderly patients with gynaecological malignancies and systematically implement related interventions [7].

The health belief model (HBM) was developed by Rosenstock [8] in the 1950s. The HBM is a framework used to motivate people to take actions that have positive health benefits, with preventing negative health consequences as a primary motivation [8, 9]. The HBM focuses on the formation of individual health beliefs by influencing patients' beliefs, guiding the formation of their health compliance behaviours, and then improving the patient's physical function status. In recent years, HBM-based interventions have received increasing clinical attention [10, 11].

Many studies [10, 11] have confirmed that HBM education interventions can improve patients' cognition of disease and improve patients' confidence and compliance with treatment. Previous evidence [12, 13] suggests that HBM-based education can improve women's perceived susceptibility to cervical cancer and perceived self-efficacy to participate in cervical cancer screening and increase screening coverage. HBM educational interventions [14] can help cancer patients fight the disease and survive longer. Other evidence [10] has also shown that an HBM-based nursing intervention can prevent the occurrence of lymphedema after breast cancer surgery, which is considered a cost-effective intervention. However, the effects of HBM education intervention on self-perception, psychological resilience, and postoperative complications in women with gynaecological malignancies, especially in elderly women with a high incidence of complications, are still unclear.

In this study, we aimed to explore the effect of perioperative HBM-based education interventions on the postoperative rehabilitation of elderly patients with gynaecological malignant tumours, providing evidence for the application of HBM-based interventions in elderly patients with gynaecological malignant tumours.

## 2. Participants and Methods

### 2.1. Participants

The present study, a randomized controlled trial, was conducted from January 2019 to August 2020. Elderly (60 years and older) women with gynaecological malignant tumours who were treated in Fujian Maternity and Child Health Hospital were included in this study. All participants were required to meet the following inclusion criteria: (1) initially diagnosed with gynaecological malignant tumours (including cervical, endometrial, and ovarian cancers) by histopathology and (2) age 60 years or older. Participants meeting the following criteria were excluded: (1) diagnosed with benign gynaecological tumour by postoperative pathology, (2) had LEDVT before the operation, (3) did not know their disease status, (4) suffered other major life events (such as divorce or widowhood) or traumatic events (such as natural disasters or man-made disasters) in the previous six months, (5) had previously had other malignancies, (6) had mental disorders or mental retardation, (7) were unable to communicate normally in the Chinese language, and (8) were lost to follow-up. All eligible participants were randomly divided into an HBM education intervention group and a basic nursing group using a randomized comparison table. We performed a sample size calculation according to two independent design data calculation formulas:

(1) $$\begin{array}{c} n_{A}=\kappa n_{B}\text{ and }n_{B}=\left(1+\frac{1}{\kappa }\right){\left(\sigma \frac{Z_{1-\alpha /2}+Z_{1-\beta }}{\mu_{A}-\mu_{B}}\right)}^{2},\\ 1-\beta =\Phi \left(Z-Z_{1-\alpha /2}\right)+\Phi \left(-Z-Z_{1-\alpha /2}\right),Z=\frac{\mu_{A}-\mu_{B}}{\sigma \sqrt{1/n_{A}+1/n_{B}}}. \end{array}$$

*κ*=*n*_*A*_/*n*_*B*_ is the matching ratio, *σ* is the standard deviation, and Φ is the standard normal distribution function. The result we obtained was that each group needed at least 63 patients. The sample size calculated was sufficient, and the power was 0.8. HBM indicators were assessed twice for all participants before and after the intervention. The data of this study came from the Hospital Information System (HIS). The HIS system is an automatic recording system of medical data generated in the process of diagnosis and treatment of patients. The HIS system can record all the treatment processes of patients, including treatment method, treatment time, treatment effect, prognosis, and follow-up. In China, the HIS system is an automatic data recording system that is purchased by the government and widely used in all government-sponsored hospitals (Figure 1). Informed consent for the research was obtained from all participants prior to the study. This study was approved by the Ethics Committee of the Fujian Maternity and Child Health Hospital (2014-068).

### 2.2. HBM Education Intervention Preparation

The intervention team consisted of 7 members: 1 head nurse, 3 gynaecological duty nurses, and 3 doctors. To ensure the effectiveness of the intervention, the head nurse arranged the intervention content and trained the nurses in a unified way so that they were familiar with the intervention content. The video “prevention of LEDVT-healthy exercise in bed” was made for the intervention group and was strictly reviewed by gynaecological clinical medicine experts and the Nursing Department of our hospital. The set of videos was composed of five episodes, including information of the following phases: before the operation, the period of anaesthesia-induced unconsciousness after the operation, and within 6 h, 7–23 h, and 24 h after waking from anaesthesia to discharge.

### 2.3. HBM Intervention Programme Implementation

According to the patient's understanding, in-person education, evaluation, guidance, and training were carried out through a combination of face-to-face teaching, video observation, simulation teaching, handgrip guidance, etc. Each session did not exceed 30 min, and family members were invited to join. The intervention programme mainly included three stages.

In the first stage (the first day after operation), the aim of the educational component was to enhance health awareness, change cognitive bias, and carry out a cognitive evaluation. The details were as follows. (1) According to the patients' own specific status, they might be given individualized psychological response education, HBM guidance, or self-coping methods. (2) After assessing the inner thoughts of the depressed patients and obtaining support and cooperation from their families, the patients were encouraged to face the disease positively and optimistically, strengthening their confidence in overcoming the disease and their educational compliance. (3) The causes, diagnosis, treatment, nursing, and postoperative complications of common gynaecological malignant tumours were explained to the patients, helping them understand the disease and correct any misunderstanding.

In the second stage (2–5 days after the operation), the aim of the educational component was to implement and evaluate the health behaviours of patients and establish a sense of self-efficacy. The details were as follows. (1) Successful experiences were shared, the patients' subjective initiative in the treatment process was encouraged, and participants were made to consciously realize that proactive health behaviour can reduce postoperative complications. (2) Patients were encouraged to actively participate in the management of their own diseases, and psychological adjustment methods such as emotional transfer and transformation, relaxation training, and discussion methods were explained and demonstrated to patients. (3) The patients were allowed to continue to watch the health exercise videos from their beds and were guided through the exercises. The individual pain threshold and psychological characteristics of patients were determined, the flow chart of the bed health exercise training plan was formulated, the purpose and method of health exercise were explained to patients and their families by the intervention nurse, and a targeted demonstration of the operation and guidance was provided to patients. (4) The patients were guided and encouraged to put the acquired knowledge into action and to play the video twice a day with “one-to-one” guidance and training assistance. The nurse often evaluated and guided the patients' rehabilitation training again, urging them to conduct the training according to the programme.

In the third stage (from the 5th day after operation to discharge), the educational theme was to implement and evaluate health education. The details were as follows. (1) Based on the theoretical framework of the HBM, questions and answers were formulated to help patients establish health beliefs and engage in healthy behaviours to promote postoperative rehabilitation. For patients with incorrect answers and training, the intervention nurse provided additional explanations and demonstrations until most of the patients answered more than 80% of the questions correctly. (2) On the day of discharge, the intervention nurse reassessed the patient's mastery of the content of healthy behaviours and patiently answered the questions raised by the patient. Further striving for the cooperation and support of relatives and society, patients were urged to continue to establish health beliefs and adopt healthy behaviours and were directed to review the material regularly and to enhance their self-care ability. (3) The nurse made a rehabilitation training plan for the discharged patients, and the family members urged the patients to complete the plan. The patients were followed up 1–2 times/week by telephone.

### 2.4. Evaluating Indicators of Intervention Effect

Indicators included compliance with training, psychological resilience, self-care ability, self-efficacy, psychological flexibility, and incidence of LEDVT. All the indicator questionnaires have been used in China, and their validity and reliability have been verified [15–19]. We once again investigated the validity and reliability of HBM index questionnaires among all our participants. To evaluate the validity, we invited 6 senior nursing physicians to carry out the item-content validity index (I-CVI) for each item using a Likert scoring system. The average I-CVI for all items was calculated as the scale-content validity index (S-CVI). The internal consistency was assessed with Cronbach's alpha coefficients of each subscale. All participants were evaluated by highly trained senior nurses twice before the intervention and one day before discharge. To ensure the consistency of the results, only one observer (senior nursing physician) was used to evaluate the indicators of all participants.

Training compliance was assessed as follows: (a) complete compliance: patients actively participated in the exercise and actively completed more than 80% of the rehabilitation exercises after being reminded. (b) Partial compliance: patients actively participated in the exercise, but they needed the supervision and inspection of nursing staff or family members to complete 31–79% of the rehabilitation exercises. (c) Noncompliance: patients did not actively participate in exercise or chose to reduce exercise time, and they completed only 30% or less of the rehabilitation exercise content. Partial compliance and noncompliance represented low compliance. Psychological resilience was assessed as follows. The Chinese version of the Connor Davidson Resilience Scale (CD-RISC) was used to assess the level of psychological resilience of patients [15]. Psychological resilience included three factors, including tenacity, strength, and optimism. The CD-RISC consisted of 25 items and was categorized into 5 levels. For each item, “0 (never) to 4 (always)” was chosen in response to the item, and the total score was 100. The self-care ability scale was used as follows [16, 17]: the scale included 11 items assessing various domains, such as self-care skills, self-concept, self-care responsibility, and self-care knowledge. Each item had a score of 0–4 points. The better the self-care ability, the higher the score. Self-efficacy was assessed as follows. The self-efficacy scale (GSE) [18, 20] was developed by the German scholar Schwarzer. There are 10 items in the GSE, with a score ranging from 1 (not at all true) to four (exactly true); a high score represents high self-efficacy. The scale has good reliability and validity in our country. Psychological flexibility was assessed as follows. The PsyFlex questionnaire [19, 21] was used to assess the psychological flexibility, including contacting the present moment, diffusion, acceptance, self-as-context, values, and committed action, of an individual (6 items, 5-point Likert scale). An example item is “Even if I am somewhere else with my thoughts, in important moments, I can focus on what is going on at that time”. Each item is scored from one (very often) to five (very seldom). The total score was reversed so that a higher score was indicative of greater psychological flexibility. The PsyFlex question items showed good internal consistency in our study sample (*α* = 0.83). The incidence of postoperative LEDVT was assessed as follows [22]. From the first day after the operation, LEDVT was evaluated daily on the patients' lower extremities, and the circumference changes at 15 cm above the patella and 15 cm below the patella were measured with a ruler to evaluate the tenderness of the gastrocnemius muscle, muscular tension, Homans sign, limb temperature, the skin colour of extremities, and pulsation of the dorsalis pedis artery. In the case of one or more abnormalities, colour Doppler ultrasonography in the double lower extremity vein was performed to determine whether LEDVT existed.

### 2.5. Statistical Analysis

Statistical analysis was performed using SPSS 20.0 software (IBM, Armonk, NY, USA). In the statistical analysis of the difference between the two groups, a normality test was first performed for the measurement data, a *T*-test was used for those with a normal distribution, and a nonparametric test was used for those with nonnormal distribution. The *X*^2^ test or Fisher's test was used to analyse the differences in enumeration data. Categorical data are expressed as percentages, and measurement data are described as the means ± standard deviations (SDs). The differences were considered statistically significant when *P* < 0.05.

## 3. Results

### 3.1. General Information of Participants

The study originally recruited 301 participants; 33 were excluded based on the exclusion criteria, and 268 eligible participants (including 137 patients with cervical cancer, 82 patients with endometrial cancer, and 48 patients with ovarian cancer) were eventually included in the study. According to the randomized comparison table, we divided 268 eligible participants into two groups: 134 women were included in the HBM education intervention group, and 134 women were included in the basic nursing group. One woman in the basic nursing group was lost to follow-up, and 133 women were eventually included in the basic nursing group analysis. We analysed the characteristics of participants between the two groups. As shown in Table 1, there were no significant differences in age (*P* = 0.603), BMI (*P* = 0.656), educational level (*P* = 0.475), marital status (*P* = 0.509), medical expenses (*P* = 0.715), tumour type (*P* = 0.755), International Federation of Gynecology and Obstetrics (FIGO) stage (*P* = 0.668), hospitalization time (*P* = 0.614), or basic venous thromboembolism (VTE) risk (*P* = 0.02) between the two groups. The I-CVI of the HBM indicator ranged from 0.82 to 0.96, and the S-CVI was 0.93. Cronbach's alpha coefficients of each subscale ranged from 0.72 to 0.93, and the values for the total score were 0.86 and 0.85 in the HBM group and control group, respectively.

### 3.2. Comparison of HBM Indicator Scores between the HBM Education Group and the Basic Nursing Group before Educational Intervention

Before the educational intervention, HBM indicator scores were compared between the two groups (Table 2), and the complete compliance of training, psychological resilience score, psychological flexibility, self-care knowledge, self-concept, self-care responsibility, self-care skills, and self-efficacy were 28.4% (38/134), 50.43 ± 3.29, 48.98 ± 3.45, 34.22 ± 7.47, 20.87 ± 4.34, 20.44 ± 4.58, 22.78 ± 6.71, and 26.49 ± 5.26, respectively. There were no differences compared to the basic nursing group (all *P* > 0.05).

### 3.3. Comparison of HBM Indicator Scores between the Two Groups after the Educational Intervention

The results in Table 3 show that after the HBM educational intervention, women in the HBM education group had higher training compliance (80.6% vs. 30.1%, *P* < 0.001), psychological resilience scores (55.47 ± 5.01 vs. 50.46 ± 2.62, *P* < 0.001), psychological flexibility scores (56.53 ± 4.51 vs. 49.13 ± 3.62, *P* < 0.001), self-care knowledge scores (43.36 ± 7.60 vs. 34.05 ± 6.99, *P* < 0.001), self-concept scores (29.57 ± 5.67 vs. 20.11 ± 3.86, *P* < 0.001), self-care responsibility scores (27.54 ± 5.09 vs. 20.86 ± 4.53, *P* < 0.001), self-care skills scores (34.51 ± 5.62 vs. 21.62 ± 5.64, *P* < 0.001), and self-efficacy scores (30.79 ± 4.56 vs. 26.41 ± 6.37, *P* < 0.001) than those in the basic nursing group. Additionally, the incidence of LEDVT decreased (2.2% vs. 8.3%, *P* = 0.027).

### 3.4. Comparison of HBM Scores between the Two Groups before and after the Intervention

In the HBM education group, women had higher training compliance (80.6% vs. 28.4%, *P* < 0.001), psychological resilience scores (55.47 ± 5.01 vs. 50.43 ± 3.29, *P* < 0.001), psychological flexibility scores (56.53 ± 4.51 vs. 48.98 ± 3.45, *P* < 0.001), self-care knowledge scores (43.36 ± 7.60 vs. 34.22 ± 7.47, *P* < 0.001), self-concept scores (29.57 ± 5.67 vs. 20.87 ± 4.34, *P* < 0.001), self-care responsibility scores (27.54 ± 5.09 vs. 20.44 ± 4.58, *P* < 0.001), self-care skills scores (34.51 ± 5.62 vs. 22.78 ± 6.71, *P* < 0.001), and self-efficacy scores (30.79 ± 4.56 vs. 26.49 ± 5.26, *P* < 0.001) after the educational intervention than before the intervention. However, there was no such change in the basic nursing group (Table 4).

## 4. Discussion

Elderly patients' cognition is relatively poor, and their psychological flexibility level is low. When confronted with disease challenges, they often cannot fully and correctly understand the disease and make reasonable and positive self-adjustments in time [23]. Gynaecological cancer surgery and postoperative life place a substantial amount of pressure on patients. When elderly patients know that they are suffering from gynaecological malignant tumours, they also experience high levels of psychological distress. Moreover, high medical costs, curative effects, and adverse reactions will also cause patients to experience fear, which leads patients to experience depression, anxiety, negative and pessimistic psychological issues, and pessimism [24]. Therefore, reasonable rehabilitation intervention based on the HBM will allow patients to develop new mechanisms of cognition and evaluation of their disease, construct new psychological defences, change their coping style, and improve their quality of life [25].

In this study, according to the characteristics of cognitive bias and a low level of psychological flexibility of elderly patients with gynaecological cancer, rehabilitation education based on the HBM and positive psychological counselling were used to improve their cognition of the disease, alleviate their negative emotions, realize their potential, and play the subjective and active role of patients in the treatment process. Moreover, by actively organizing and continuously guiding patients to perform health exercise training in bed, we consolidated and deepened patients' grasp of intervention information and skills, which allowed patients to gradually establish a positive psychological state and actively participate in and cooperate with rehabilitation treatment. Our results indicated that the level of psychological resilience of elderly patients with gynaecological cancer was significantly increased after rehabilitation based on the HBM, which suggested that rehabilitation based on the HBM was an important measure to improve the psychological resilience of patients with gynaecological cancer. Rehabilitation based on the HBM can enhance the psychological resilience and rehabilitation compliance of patients, leading patients to actively participate in postoperative rehabilitation treatment and achieve a more ideal rehabilitation effect. Previous studies [26, 27] have also shown that psychological interventions can improve survival in cancer patients. This evidence further proves the value of HBM psychological intervention in elderly gynaecological cancer patients in improving survival.

There is likely to be a certain correlation between physical health and treatment compliance. Early psychological intervention can improve treatment compliance in cancer patients [28]. Patients with a high level of mental flexibility and good mental health are able to actively participate in and cooperate with treatment, so they have higher compliance with rehabilitation training [29]. Our study shows that the level of patients' psychological resilience and compliance can be increased through positivity HBM education. HBM education can help patients face their disease positively, rebuild their confidence, adopt healthy behaviours, and enhance their psychological immunity, increasing their level of psychological resilience [25].

Self-efficacy is an important factor in maintaining or changing health behaviours. The higher the level of self-efficacy, the higher the level of adopting, maintaining, and striving for healthy behaviours and the stronger the self-nursing ability [30]. According to Wen Y's [31] study, the early self-nursing ability of patients affects later outcomes. Therefore, perioperative rehabilitation education based on the HBM can not only strengthen the self-nursing ability of patients with malignant tumours but also increase the self-nursing ability and quality of life after discharge.

The decline in the learning and memory abilities of elderly patients can impact their self-efficacy and self-nursing abilities. In the context of special diseases, patients can build and strengthen their self-efficacy and self-nursing skills only through active intervention, reconstruction of their self-confidence to overcome difficulties, and continuous demonstrative learning [32]. In light of the decline in learning and memory ability of elderly patients with gynaecological malignant tumours, during HBM-based health education, the patients were trained in the diaphragm and lower extremity movements through the guidance of professional nurses and video demonstrations and were supervised in the hospital and during follow-up after discharge in this study. The results indicated that the self-efficacy and self-nursing ability in the intervention group were much higher than those in the control group after the application of rehabilitation education based on the HBM, suggesting that rehabilitation education based on the HBM can help elderly patients with gynaecological cancer master disease-related knowledge and skills, enhance their self-efficacy, adopt good rehabilitation behaviour and self-nursing ability, and improve rehabilitation.

LEDVT is one of the most common complications in gynaecological patients [33]. It can cause pain, swelling, and dysfunction of the lower limbs. Thrombus detachment of LEDVT can induce pulmonary embolism and is even life-threatening. Elderly patients with gynaecological cancer require a wide range of operations, a long duration of bed rest after the operation, and a low willingness to perform activities due to lower limb dysfunction. Moreover, elderly patients with gynaecological cancer have high-risk factors, such as old age, malignant tumours, and other vascular diseases [33], which makes the probability of LEDVT higher than that among general patients. Based on the individual differences in elderly patients with gynaecological malignant tumours, rehabilitation intervention based on the HBM can help patients fully understand the mechanism and severity and the importance of cooperative treatment and health exercise training for LEDVT and enhance their health beliefs and active participation consciousness. Postoperative rehabilitation training can effectively reduce the occurrence of deep vein thrombosis (DVT) [34]. One-on-one guidance from the intervention nurse can promote the patients' transition from passive exercise to active routine exercise, improve the prognosis of patients, and effectively reduce the incidence of LEDVT [22]. The results of this study showed that the incidence of LEDVT in elderly patients with gynaecological cancer decreased significantly after receiving HBM-based rehabilitation education, indicating that strengthening HBM rehabilitation interventions can promote the postoperative rehabilitation of elderly patients with gynaecological cancer, especially by effectively preventing LEDVT.

There are still some potential limitations to this study. First, the number of participants in this study was small, and we will add more participants in the next stage to further verify the effectiveness of the HBM education intervention. Second, this study was conducted in a single centre, and the reproducibility of the results is still unclear, so it will be extended to multiple centres to verify the applicability of the HBM in the future. Finally, the follow-up data of the participants were not analysed in this study because our follow-up work is ongoing, and we will analyse the results after the follow-up is completed.

## 5. Conclusion

Evidence from this study suggests that perioperative HBM-based educational interventions benefit mental health and disease outcomes in elderly women with gynaecological malignancies by improving self-efficacy, self-care ability, and compliance.

## Figures and Tables

**Figure 1:** Flowchart of this study. HBM, health belief model.

**Table 1:** Comparison of individual characteristics in the two groups.

Characteristics	HBM education group (*n* = 134)	Basic nursing group (*n* = 133)	*P* value
Age (years, ±SD)	66.90 ± 7.25	67.35 ± 6.86	0.603
BMI (±SD)	24.77 ± 3.29	24.58 ± 3.45	0.656

*Educational level (n (%))*			
≤ junior middle school	98 (73.1)	92 (69.2)	0.475
≥ senior high school	36 (26.9)	41 (30.8)	

*Marital status (n (%))*			
Married	112 (83.6)	115 (86.5)	0.509
Unmarried	22 (16.4)	18 (13.5)	

*Medical expenses (n (%))*			
Medical insurance	118 (88.1)	119 (89.5)	0.715
Self-paying	16 (11.9)	14 (10.5)	

*Tumour types (n (%))*			
Cervical cancer	66 (49.3)	71 (53.4)	0.755
Endometrial cancer	42 (31.3)	40 (30.1)	
Ovarian cancer	26 (19.4)	22 (16.5)	

*FIGO stages (n (%))*			
I	66 (49.3)	69 (51.9)	0.668
≥II	68 (50.7)	64 (48.1)	

*Hospitalization times (n (%))*			
<3	126 (94.0)	123 (92.5)	0.614
≥3	8 (6.0)	10 (7.5)	

*Basic VTE risk (n (%))*			
Middle risk	56 (41.8)	61 (45.9)	0.502
Extremely high risk	78 (58.2)	72 (54.1)	

HBM, health belief mode; SD, standard deviation; FIGO, International Federation of Gynecology and Obstetrics; VTE, venous thrombus embolism.

**Table 2:** Comparison of HBM indicator scores between the HBM education group and the basic nursing group before educational intervention.

Variables	HBM education group (*n* = 134)	Basic nursing group (*n* = 133)	*P* value
*Compliance of training*			
Complete compliance (n (%))	38 (28.4)	37 (27.8)	0.922
Low compliance (n (%))	96 (71.6)	96 (72.2)	

Psychological resilience score ($\bar{\text{x}}$±SD)	50.43 ± 3.29	50.55 ± 2.29	0.738
Psychological flexibility ($\bar{\text{x}}$±SD)	48.98 ± 3.45	49.29 ± 3.59	0.465
Self-care knowledge ($\bar{\text{x}}$±SD)	34.22 ± 7.47	33.77 ± 7.05	0.614
Self-concept ($\bar{\text{x}}$±SD)	20.87 ± 4.34	20.22 ± 4.10	0.206
Self-care responsibility ($\bar{\text{x}}$±SD)	20.44 ± 4.58	20.64 ± 4.71	0.727
Self-care skills ($\bar{\text{x}}$±SD)	22.78 ± 6.71	21.77 ± 5.82	0.190
Self-efficacy ($\bar{\text{x}}$±SD)	26.49 ± 5.26	26.29 ± 6.41	0.781

HBM, health belief model; $\bar{\text{x}}$, mean; SD, standard deviation.

**Table 3:** Comparison of HBM indicator scores between the two groups after the educational intervention.

Variables	HBM education group (*n* = 134)	Basic nursing group (*n* = 133)	*P* value
*Compliance of training (n (%))*			
Complete compliance	108 (80.6)	40 (30.1)	<0.001
Low compliance	26 (19.4)	93 (69.9)	

Psychological resilience score ($\bar{\text{x}}$±SD)	55.47 ± 5.01	50.46 ± 2.62	<0.001
Psychological flexibility ($\bar{\text{x}}$±SD)	56.53 ± 4.51	49.13 ± 3.62	<0.001
Self-care knowledge ($\bar{\text{x}}$±SD)	43.36 ± 7.60	34.05 ± 6.99	<0.001
Self-concept ($\bar{\text{x}}$±SD)	29.57 ± 5.67	20.11 ± 3.86	<0.001
Self-care responsibility ($\bar{\text{x}}$±SD)	27.54 ± 5.09	20.86 ± 4.53	<0.001
Self-care skills ($\bar{\text{x}}$±SD)	34.51 ± 5.62	21.62 ± 5.64	<0.001
Self-efficacy ($\bar{\text{x}}$±SD)	30.79 ± 4.56	26.41 ± 6.37	<0.001

*Incidence of LEDVT (n (%))*			
Yes	3 (2.2)	11 (8.3)	0.027
No	131 (97.8)	122 (91.7)	

HBM, health belief model; $\bar{\text{x}}$, mean; SD, standard deviation; LEDVT, lower extremity deep vein thrombosis.

**Table 4:** Comparison of HBM scores between the two groups before and after intervention.

Groups	Variables	Before intervention	After intervention	*P* value
HBM education group (*n* = 134)	*Compliance of training (n)*			<0.001
	Complete compliance	38	108	
	Low compliance	96	26	
	Psychological resilience score ($\bar{\text{x}}$±SD)	50.43 ± 3.29	55.47 ± 5.01	<0.001
	Psychological flexibility ($\bar{\text{x}}$±SD)	48.98 ± 3.45	56.53 ± 4.51	<0.001
	Self-care knowledge ($\bar{\text{x}}$±SD)	34.22 ± 7.47	43.36 ± 7.60	<0.001
	Self-concept ($\bar{\text{x}}$±SD)	20.87 ± 4.34	29.57 ± 5.67	<0.001
	Self-care responsibility ($\bar{\text{x}}$±SD)	20.44 ± 4.58	27.54 ± 5.09	<0.001
	Self-care skills ($\bar{\text{x}}$±SD)	22.78 ± 6.71	34.51 ± 5.62	<0.001
	Self-efficacy ($\bar{\text{x}}$±SD)	26.49 ± 5.26	30.79 ± 4.56	<0.001

Basic nursing group (*n* = 133)	*Compliance of training (n)*			0.685
	Complete compliance	37	40	
	Low compliance	96	93	
	Psychological resilience score ($\bar{\text{x}}$±SD)	50.55 ± 2.29	50.46 ± 2.62	0.467
	Psychological flexibility ($\bar{\text{x}}$±SD)	49.29 ± 3.59	49.13 ± 3.62	0.124
	Self-care knowledge ($\bar{\text{x}}$±SD)	33.77 ± 7.05	34.05 ± 6.99	0.076
	Self-concept ($\bar{\text{x}}$±SD)	20.22 ± 4.10	20.11 ± 3.86	0.527
	Self-care responsibility ($\bar{\text{x}}$±SD)	20.64 ± 4.71	20.86 ± 4.53	0.181
	Self-care skills ($\bar{\text{x}}$±SD)	21.77 ± 5.82	21.62 ± 5.64	0.519
	Self-efficacy ($\bar{\text{x}}$±SD)	26.29 ± 6.41	26.41 ± 6.37	0.404

HBM, health belief model; $\bar{\text{x}}$, mean; SD, standard deviation.

## Data Availability

The data used to support the findings of this study are available from the corresponding author upon request.
